# Improved On-Demand Travel Route Planning Model with Interest Fields

**DOI:** 10.1155/2022/6442441

**Published:** 2022-08-09

**Authors:** Limin Yan

**Affiliations:** Zhengzhou University of Science and Technology, Zhengzhou 450000, China

## Abstract

Intelligent tourism route planning is an important element of smart tourism, and the current tourism route planning has problems such as strong subjectivity and low personalization considering tourists' interests. To solve the problems of current tourism route planning, an improved interest field travel route planning model is proposed. Firstly, an intelligent interest field extraction model is established. Secondly, an improved greedy algorithm is designed to reduce the risk of missing the optimal solution, strengthen the local search capability, and improve the solution accuracy of the algorithm. The extracted routes of interest sites are planned, and a motivated iterative value output model is established. The experimental results demonstrate that the selected routes are shorter and less expensive than the traditional model. By iterating the actual data to obtain the iterative values of different tourist route motivations and the sequential guide map of attractions based on tourist interests, the optimal and suboptimal routes that satisfy the tourist motivation interests are analyzed. This model has strong feasibility and practical significance for smart tourism route planning.

## 1. Introduction

With the continuous improvement of people's living conditions, tourism has been gradually developed, and travel has become a favored form of leisure. Tourists release their inner stress, taste food, and enjoy the beautiful scenery in this manner [1]. The tourist route chosen is a significant consideration that should be considered prior to travel [2, 3]. Optimizing the tourist route can reduce the cost of travel, improve the efficiency of tourism, and ensure that people enjoy a better experience in tourism [4, 5]. At present, the design of tourism routes adheres to the concept of “freedom, individuality, exploration, and mastery.” Based on these design concepts, the original itineraries need to be properly optimized to ensure the growing tourist purposefulness [6]. The original tourism route optimization model has a poor linkage between tourism route factors when optimizing tourism routes, resulting in the problem of poor shortest route selection.

The tourism route planning problem is based on the evolution of the classical traveler problem, whose main idea is to optimize the combination of attractions of candidate cities, according to certain rules [7]. This problem has been studied quite extensively at home and abroad, and other better techniques for this issue have already been developed, including the dynamic programming method [8] and simulated annealing algorithm [9]. The literature [10] provides a multiobjective route planning method for bicycle travel by considering the factors of time, expense, and service. The literature [11] proposed an improved hybrid frog-hopping algorithm for the problem of slow iteration of the frog-hopping algorithm, which improved the evolution speed and accuracy of the algorithm, and used it to optimize the parameters of the artificial potential field to improve the path planning capability. In the literature [12], a meta-heuristic-based approach is proposed to better guide the search process by integrating a biased randomization strategy within a variable neighborhood search framework. The method is used to solve a multisite vehicle path problem that simultaneously considers economic, environmental, and social dimensions. The literature [13] proposed an improved A^*∗*^ algorithm for the scenic path planning problem, which effectively improves the computational efficiency and reduces the road cost. The literature [14] dynamically obtains the optimal path through the remaining attractions and remaining paths in the scenic area. The literature [15] uses the weight matrix road to improve the ant colony algorithm and constructs the optimal path planning model. The literature [16] introduces attributes such as interest points into the attention and deep learning model to achieve flexible path planning. The method uses a fuzzy C-mean clustering method [17] to cluster information in intelligent tourist route planning and performs tourist route planning at the center of the clusters.

Among the existing conventional tourism route planning methods, the distributed scheduling method using association rules can mine tourist behavior information for intelligent tourism route planning to improve the accuracy of planning [18]. However, the method has a high statistical overhead and high cost. The recommendation method using joint information entropy features of tourist preferences and tourist routes is also commonly used [19], but its recommendation accuracy is low when used for large-scale tourist route recommendations. Tourist route planning models using heuristic optimization algorithms are not high enough in optimization performance. The modeling time of travel route planning methods using deep learning models is long [20]. In addition, these existing algorithms tend to ignore the problem of users' interests and needs in the middle of tourism trips.

Before visiting a tourist city, tourists usually plan their travel routes based on their interest points, the types and characteristics of attractions in the city, and the facilities around the attractions to obtain the maximum motivational benefit in a limited time. They have a direct impact on the distribution of interest fields, types of interest fields, and specific tourist routes, respectively [21]. At present, tourism GIS is mainly developed for mass tourism services, providing a large amount of tourism geographic information for tourists to query and analyze. The degree of personalization of mass tourism geographic information services is low, especially when travelers are less familiar with the tour cities, and it is difficult to obtain the maximum motivational benefit by subjective planning of tourist routes. Therefore, determining the best tourist route according to the tourist's interest demand is an important research direction of personalized tourism and an important element of tourism GIS development and smart tourism service [22]. It contributes significantly to the city's tourism fever, enhancing the image of the city, expanding the influence of city tourism, and enhancing the development of the city tourism business. City attractions can be divided into several categories according to their nature, and for a particular attraction, the tourist group's interest in tourism and its evaluation of the attraction are important factors that influence subsequent tourists to choose the attraction and plan the tourist route [23].

In this paper, based on the above research, an improved on-demand travel route planning model with interest fields is proposed. The proposed model uses an improved iterative algorithm to plan the best tourist routes based on the interest needs of tourist individuals or groups. The proposed model is validated by simulation using actual tourist attractions and data as an example of the tourist route optimization problem. The proposed model can determine the optimal tourist route solution and provide supplementary decision support for tourists' travel.

The innovations and contributions of this paper are as follows:

1. The algorithm model of this paper establishes the interest field model of urban attractions and determines the distribution of statistical sample interest attractions.
2. An improved greedy algorithm introducing a two-way search algorithm and ant colony algorithm is designed.
3. The shortest path between attractions is determined by the improved greedy algorithm, and the motivated iterative value output model is established.
4. The optimal travel route plan is determined according to the interest demand of travel individuals or groups.

This paper consists of four main parts: the first part is introduction, the second part is methodology, the third part is result analysis and discussion, and the fourth part is conclusion.

## 2. Methodology

### 2.1. Interesting Spots Model

The city's overall type and number of representative tourist attractions are determined, and the feature coding set of city attractions is constructed first. The interests are classified according to different attributes, and the subset of attraction feature codes is built. The attraction feature codes contained in the subset are the attraction feature code elements. The attraction feature coding set is an important data source for tourism subjects' intelligent random selection of attractions. The choice of attraction feature coding subsets and attraction coding elements by calling random functions is the way to achieve brilliant or manual selection.

Attraction feature coding set: define the total set of city attractions coded by all representative attractions of the city and their collections as the feature coding set *P* and its subsets as the feature coding subsets.

Attraction feature encoding subset: define the set of urban attractions coded by a representative class of attractions and their elements as the subset of attraction features coded by *P*_*x*_. Where *x* ∈ (0, *n*] ⊂ **Z**^+^ and *n* is the number of urban attraction categories satisfying *n* ∈ (0, *n*_max_] ⊂ **Z**^+^. *P*={*P*_*x*_*|x* ∈ (0, *n*] ⊂ **Z**^+^}.

Attraction feature code element: define the unique feature code of each attraction as the attraction feature code element.

Let the attraction feature subunit **P**_*x*_ contain *e*_*x*_ attraction feature codes, and then the total number of attraction feature code set elements is ∑_*x*=1_^*n*^*e*_*x*_. Let the elements of attraction feature codes in ∀**P**_*x*_ be *P*_*x*_*Q*_*y*_, and *y* ∈ (0, *e*_*x*_]. Define the 1 × *e*_*x*_ dimensional vector **P**_*x*_ consisting of ∀**P**_*x*_ elements as the base vector of the attraction feature encoding subset, and then there is *P*_*x*_=[*P*_*r*_*Q*_1_, *P*_*r*_*Q*_2_,…, *P*_*r*_*Q*_*e*_*x*__]. The *n* × max*e*_*x*_ dimensional subunit matrix **U** is constructed by taking the maximum value of the vertical column dimension max*e*_*x*_. The matrix arranges the base vectors **P**_*x*_ in the order of least to most elements in the attraction feature coding subset, and zeroes complement the deficiencies. There is formula (1), which constitutes the attraction feature coding set matrix.

(1) $$\begin{array}{c} U=\left[\begin{array}{c} \begin{array}{cccccc} P_{1}Q_{1} & P_{1}Q_{2} & \ldots & P_{1}Q_{e_{1}} & 0 & 0 \end{array}\\ \begin{array}{cccc} P_{2}Q_{1} & P_{2}Q_{2} & P_{2}Q_{e_{2}} & 0 \end{array}\\ \begin{array}{cc} \vdots & \vdots \end{array}\\ \begin{array}{cccc} P_{n}Q_{1} & P_{n}Q_{2} & \ldots & P_{n}Q_{\text{max}e_{x}} \end{array} \end{array}\right]. \end{array}$$

The uniform distribution function *I* ~ *F*(*g*, *h*) on [*g*, *h*] is chosen as the intelligent random number generator. Suppose the tourist leaves it entirely to the intelligent machine to randomly select the attractions. It is sufficient to provide the number of demand types *w* and the number of attractions *t*_*r*_ for each demand type. Where *w* ∈ (0, *n*], *r* ∈ (0, *w*], *t*_*r*_ ∈ (0, *e*_*x*_]. The smart machine first calls the uniform distribution function on [1, *n*] to extract m attraction types, and then each calls the uniform distribution function on [1, *e*_*x*_] to generate *t*_*r*_ attraction codes, with a total of *t* = ∑_*r*=1_^*w*^*t*_*r*_ attraction codes. If the tourist selects the attraction independently, then *w* and *t*_*r*_ can be determined directly. Then the combination of demanded attraction types in *C*_*n*_^*w*^ and the various types of demanded attraction types are *C*_*e*_*x*__^*t*_*r*_^.

#### 2.1.1. Feature Interest Sites

The n attractions selected randomly by the smartphone or directly by the tourist subject are defined as the feature interest attractions. The feature interest sites are the sites selected by the tourist subject that best meet the subject's psychological needs and can be visited in a limited amount of time.

#### 2.1.2. Feature Attraction Priority

The priority of a feature attraction is defined as the level of interest of the tourist subject in the feature attraction. The higher the intensity of interest is, the more attractive the attraction is to the tourist, and the more priority is given to the attraction.

### 2.2. Improved Algorithm

The raster approach is applied to model the tourism region in this article. The raster method is a technique for modeling an area that employs a sequence of grid. The raster method is utilized to build a 10 × 10 water model, see Figure 1. In Figure 1, white grids are feasible grids, representing feasible areas. Black grids are infeasible grids, representing infeasible areas, that is, the area has obstructions to navigation. Visitors cannot pass safely. The black dot in the lower left corner indicates the visitor's current position. The square in the upper right corner indicates the position the visitor needs to reach. The serial number of the grid indicates the grid coordinates. For example, the grid coordinates of the first row and column are (0, 0), and the grid coordinates of the first row and column are (0, 1). When the visitor is in any grid in the model except the edge of the model, there should be eight grids around it, and the visitor can move to any feasible grid around it.

After modeling the area with the raster method, the more complex working environment of the visitor is transformed into a simple one. The visitor's path planning problem is also transformed into the problem of finding the optimal path between two raster points.

A greedy algorithm chooses the best option for each stage, ensuring that the final result is the best overall. For example, in a backpack problem, selecting the item with the highest unit value to fill the backpack each time is a greedy algorithm. If a problem can be solved using a greedy algorithm, then in general, the greedy algorithm will be the best way to solve the problem. Greedy algorithms are often used as auxiliary algorithms or directly to solve simple issues because of their efficiency and the fact that the results obtained are close to the optimal results. The location of the visitor is presented in Figure 2.

As shown in Figure 2, the visitor is in grid 0. If all eight grids around the visitor are feasible, then all eight grids are reachable by the visitor in the next step. If there are infeasible grids among the eight grids, these grids must be removed before the next calculation step. After finding all the next reachable grids, the distance between grid *i* and the target grid end is calculated.

(2) $$\begin{array}{c} D_{x}=\begin{array}{c} \sqrt{{\left(i_{\text{end}}-i_{x}\right)}^{2}+{\left(j_{\text{end}}-j_{x}\right)}^{2}}\\ x=0,1,2,\ldots ,t, \end{array}, \end{array}$$

where *i*_end_ and *j*_end_ denote the horizontal and vertical coordinates of raster end. *i*_*x*_ and *j*_*x*_ denote the horizontal and vertical coordinates of raster *x*. *D*_0_ indicates the distance between raster 0 (where the visitors are located) and the raster end.

The closest grid to the grid end is selected from all feasible grids; that is, the grid that satisfies the condition min{*D*_1_, *D*_2_,…, *D*_*t*_} < *D*_0_ is the grid that the visitor reaches next. If no grid satisfying this condition is found, the algorithm falls into a state of local convergence and cannot continue the search.

If there are two grids *g* and *h* (*g*, *h*=0,1,2,…, *t*, *g* ≠ *h*) satisfying *D*_*a*_=*D*_*b*_; that is, when a visitor encounters a “fork in the road” during route selection, he or she generally makes a random choice for the next calculation and records the total distance of the route. Finally, the shortest path is retained by iterating several times.

The traditional greedy algorithm converges quickly and is computationally tiny, but once the algorithm falls into a state of local convergence, it cannot get out of it by itself. Therefore, it is not always possible to find the optimal path between the starting point and the end point even after conducting multiple experiments.

When a visitor moves to a grid that is not the end point during the path search, the algorithm cannot continue when it cannot find the next grid that satisfies the condition, and such problems are known as local convergence problems.

The most common local convergence problem is shown in Figure 3. When the visitor moves from grid 7 to the target point, the greedy algorithm calculates that moving to grid 0 is the optimal solution. When the visitor moves to grid 0, it is found that the element smaller than *D*_0_ cannot be found from the set {*D*_1_, *D*_5_, *D*_6_, *D*_7_, *D*_8_} by calculation. After the visitor arrives at grid 0, no optimal solution can be seen that can carry out the following analysis, and the path search comes to a standstill and the local convergence problem appears.

In fact, in the process of path search using the greedy algorithm, as long as there is a concave obstacle region in the tourist's forward direction, the possibility of the algorithm falling into a state of local convergence is high. The solution to this type of problem is mainly to add the raster where the tourist is at this time to the taboo table. Grid 0 in Figure 3 is converted from a feasible grid to an infeasible grid to prevent visitors from entering the grid again. Although the method of adding a taboo table is effective, the path search must be restarted from the origin after converting a feasible raster to an infeasible raster. This will increase the number of operations and slow down the speed of the algorithm to find the final solution.

For this type of local convergence problem, this paper introduces the two-way search algorithm in combination with the characteristics of the greedy algorithm. The two-way search algorithm runs with two directions of search simultaneously. One is the forward search from the initial to the target point, and the other is the reverse search from the target to the initial point. The search can be stopped when the paths obtained from the two directions meet in the middle or partially overlap.

The path search of the traditional greedy algorithm is a forward search from the initial to the target point. The two-way search algorithm adds a reverse search from the target to the initial point on top of the forward search. After the search stops, the forward search path is combined with the reverse search path to obtain the final path planning result for the visitor. This method is used to search the path of a randomly generated 10 × 10 area model, and the results are shown in Figure 4.

Figure 4(a) shows the results calculated by the conventional greedy algorithm. When the visitors move to the grid with coordinates (4, 6), there is no feasible grid around it that satisfies “the distance between the target grid < the distance between the grid with coordinates (4, 6) and the target grid,” and the movement of the visitors is stalled, and the algorithm is interrupted.  Figure 4(b) shows the calculation results after introducing the two-way search algorithm into the traditional greedy algorithm. The forward search result of the two-way search algorithm is the same as that of the traditional greedy algorithm, and the path obtained from the reverse search meets the path obtained from the forward search at the grid with coordinates (5, 4). The final path planning result can be obtained by combining the paths obtained from forward and reverse search.

Through several experiments, it can be seen that the introduction of the two-way search algorithm in the traditional greedy algorithm not only affects the complexity of the algorithm but also solves most of the local convergence problems and dramatically accelerates the convergence speed of the algorithm.

However, the two-way search greedy algorithm cannot produce results when there are concave obstacle areas on both forward and reverse search paths. In this scenario, the problem should be solved by the taboo table. Here, an index *X*_*wt*_ is specified for the raster with coordinates (*w*, *t*) in the area model.

(3) $$\begin{array}{c} X_{wt}=\left\{\begin{array}{cc} 1, & \text{Ant prefers the grid,}\\ \text{0,} & \text{Prohibit ants to select the grid.} \end{array}\right. \end{array}$$

*X*_*wt*_ represents the concentration of ant pheromone in the grid with coordinates (*w*, *t*), where 1 is the highest and 0 is the lowest. After the calculation, the pheromone concentration in the next optimal raster calculated by the greedy algorithm is changed to 1. The purpose of this setting is to accelerate the search speed of the ants in the next iteration. When the forward and reverse search paths cannot meet in the two-way search, and the algorithm falls into local convergence (as shown in Figure 5), the ant pheromone concentration in the raster in which the visitors is located changes as follows:

(4) $$\begin{array}{c} X_{wt}=1\Rightarrow X_{wt}=0. \end{array}$$

The raster in which the visitors on the forward and reverse search paths are located is converted from a feasible raster to an infeasible raster when local convergence occurs. The algorithm then starts the second two-way search. In this search, the visitor does not enter the raster where the local convergence occurred in the initial search but jumps out of the constraint to find a more optimal path. The two-way search greedy algorithm before and after the combination with the ant colony algorithm is provided in Figure 5.

In Figure 5(a), the forward and reverse searches fall into local convergence at the grid with coordinates (7, 2) and (3, 6), respectively, and the search is aborted. At the beginning of the second search, these two grids have been changed to an infeasible grid (as shown in Figure 5(b)). The second search avoids the raster where the local convergence occurred in the first search and successfully finds a new optimal path, with the forward and reverse search paths meeting at the raster with coordinates (4, 3).

In summary, the greedy algorithm, which combines the advantages of the two-way search algorithm and ant colony algorithm, essentially reduces the computational effort and accelerates the convergence speed of the algorithm. It also solves most of the path-finding problems in less complex environments. This improved algorithm can be used for the global path planning of tourists.

### 2.3. Modeling of Interest Spot Route Planning Algorithm

The tourist makes a one-way non-repetitive visit to the selected *t* sites of characteristic interest in a limited sufficient time. There are *G*_*t*_^*t*^ kinds of different touring orders without considering the priority of interests, and different touring orders satisfy the tourist's psychological needs to various degrees. The degree of satisfaction of motivational interests is determined quantitatively. The intelligent machine determines the best and second-best routes to satisfy the motivational interests by quantitatively iterating the output values of different tour routes and ranking them. First, in the case of interest, the tourists' randomly selected or directly selected attractions of interest can determine no more than *G*_*t*_^*t*^ tour order. The route of most interest to the tourist may be the nonintelligent machine optimal route. From the perspective of path minimization alone, the traveler goes through *t* − 1 intervals from the 1st feature interest site to the nth feature interest site. Every stretch is made out of various street nodes. The tour sequence consisting of *t* − 1 intervals has an ordered arrangement of the shortest paths, but the shortest paths output does not have the highest motivated iterative values. Considering the objective factors in the tour process, the motivation iteration value is outputted by iterating over a finite sequence of the shortest paths.

Attraction route motivation interval *B*(1, *U*_*t*_): the one-way motivation interval formed by the tour from the starting feature interest attraction 1 to the ending feature interest attraction *U*_*t*_.

Define the attraction route motivation subinterval Δ*B*_*z*_(*U*_*z*_, *U*_*z*+1_): the one-way motivation subinterval is formed by the tour of the feature interest attraction ∀*U*_*z*_ to the feature interest attraction *U*_*z*+1_. Where *z* ∈ (0, *t* − 1]. The attraction route motivation subinterval outputs the attraction route motivation iteration metric Δ*A*_*z*_(*U*_*z*_, *U*_*z*+1_). Δ*A*_*z*_(*U*_*z*_, *U*_*z*+1_) is the iteration metric of *A*(1, *U*_*t*_) that determines the final output value of *A*(1, *U*_*t*_).

Define the attraction route motivation iteration value *A*(1, *U*_*t*_): the initial value of the motivation iteration and the iterative algorithm in the attraction route subinterval Δ*B*_*z*_(*U*_*z*_, *U*_*z*+1_) is iteratively calculated and finally outputs the motivation value in the whole attraction route motivation interval *B*(1, *U*_*t*_) iteratively. The *A*(1, *U*_*t*_) value determines the magnitude of the motivation benefit and the degree of satisfaction of the motivation benefit obtained by the tourist after this attraction is selected by the intelligent machine or chosen independently.

Consider the interval between attraction ∀*U*_*z*_ and attraction *U*_*z*+1_, that is, the local interval of the whole tour route. In terms of time-saving, travel convenience, and congestion avoidance, tourists need to choose an optimal access route from sightseeing spot *U*_*z*_ to sightseeing spot *U*_*z*+1_. The ferry distance *μ*_1_, bus and subway routes *μ*_2_, cab fare *μ*_3_, number of traffic lights *μ*_4_, and congestion index *μ*_5_ are the important indicators to determine the best access route. According to the improved greedy algorithm, ∀Δ*B*_*z*_(*U*_*z*_, *U*_*z*+1_) and Δ*B*_*z*′_(*U*_*z*′_, *U*_*z*′+1_) are mutually exclusive and independent, and ∀Δ*A*_*z*_(*U*_*z*_, *U*_*z*+1_) and Δ*A*_*z*′_(*U*_*z*′_, *U*_*z*′+1_) are mutually exclusive and independent. The ferrying distance *μ*1 is determined by depth search superposition and binomial tree heap sorting, and the different access interval indicators *μ*_2_ ~ *μ*_5_ are then determined under this condition. The iterative value of attraction route motive *A*(1, *U*_*t*_) is calculated below.

**Step 1 .**

Determine the set of key road nodes *Q* within the attraction route motivation subinterval Δ*B*_*z*_(*U*_*z*_, *U*_*z*+1_). All major road nodes *v*_*q*_ between feature interest attractions *U*_*z*_ and *U*_*z*+1_ constitute the set of road nodes, where *q* ∈ (0, *q*_max_] ⊂ *Z*^+^.

**Step 2 .**

Determine the depth search overlay layer. Based on the radius *R* of the attraction *U*_*z*_ buffer and the average proximity distance between nodes $\bar{s}\left(v_{q},v_{q+1}\right)$, the set of road nodes is divided into several subsets *Z*_*h*_, *h* ∈ (0, *h*_max_], and the subsets are used as depth search layers.  Figure 6 shows spot buffer depth search overlay layer.

**Step 3 .**

Layer-by-layer depth search overlay. Let the distance between the attraction *U*_*z*_ and the *λ*th road node *v*_*λ*_ in the buffer *R*_1_ be *s*(*U*_*z*_, *v*_*λ*_), *λ* ∈ (0, *q*_max_]. The distance between ∀*v*_*λ*_ in the buffer ∀*R*_*δ*_ and its neighbor ∀*v*_*λ*′_ in ∀*R*_*δ*+1_ is *s*(*U*_*δ*_*v*_*λ*_, *U*_*δ*+1_*v*_*λ*′_). The road node interval distance stacking table is constructed as shown in Figure 7 (arrow direction is the depth direction of the search stacking distance). Construct the base vector **S**_*m*_. Let *R*_*δ*_ layer contain *λ*_*δ*_ road nodes *v*, and then there are *γ* pathway distances between attractions *U*_*z*_ and *U*_*z*+1_. Satisfying the dimension 1 × *γ* of the base vector **S**_*w*_ of the interval distance heap ordering of attractions, we have formulas (5) and (6). According to (6), we determine the inter-site distance heap sorting basis vector **S**_*w*_ as [*s*_1_, *s*_2_,…, *s*_*γ*_].

(5) $$\begin{array}{c} q_{\text{max}}=\sum_{\delta =1}^{\delta_{\text{max}}}\lambda_{\delta }, \end{array}$$

(6) $$\begin{array}{c} \gamma =\prod_{\delta =1}^{\delta_{\text{max}}}\lambda_{\delta }. \end{array}$$

**Step 4 .**

Construct a *b*-layer complete binary tree with the elements of the interval distance heap sorting base vector **S**_*m*_ in order from left to right, and determine its element positions in Figure 8. *k* in the elements *c*_*k*,*ε*_ is the layer where the element is located, satisfying *k* ∈ (0, *b*]. *ε* is the position of the element in the layer, satisfying *ε* ∈ (0, 2^*k*−1^].

Compare the *k* th level child node element bit *c*_*k*,*ε*_ with the upper-level *k* − 1 level child node element *c*_*k*−1,*ε*′_ and its subordinate *k*+1 level child node element *c*_*k*+1,*ε*′_. The jump command in Step 2 generally acts on the last node.

1. If the element bit element *c*_*k*,1_ < *c*_*k*−1,1_, then replace *c*_*k*,1_ with *c*_*k*−1,1_ both position element *s*.
2. If the element bit element *c*_*k*,1_ ≥ *c*_*k*−1,1_, keep the position element *s* of both *c*_*k*,1_ and *c*_*k*−1,1_ unchanged. If *c*_*k*−1,1_ contains only a single node, skip Step 5. If it is not a single node, continue to Step 3.
3. If the element bit element *c*_*k*,1_ < *c*_*k*−1,2_, then replace *c*_*k*,1_ with *c*_*k*−1,2_ both position element *s*.
4. If the element bit element *c*_*k*,1_ ≥ *c*_*k*−1,2_, keep *c*_*k*,1_ and *c*_*k*−1,2_ both position element *s* unchanged.
5. Return to Step 1, and keep looking for the next node *c*_*k*,2_.
6. Search to the element bits of the last child node *c*_*k*,*ε*max_ of layer *k*, complete the layer search.
7. Continue the search for other layers of child/parent nodes, traversing layers 1 to *b*. And finally, form ∀*c*_*k*,*ε*_ is greater than its previous layer child node *c*_*k*−1,*ε*′_, and the search is completed.
8. After the search is completed, the elements *c*_*k*,*ε*_ and *c*_*k*,*ε*′_ are compared, and all elements in the same layer are traversed. Let *ε* < *ε*′, if *c*_*k*,*ε*_ < *c*_*k*,*ε*′_, do not replace *c*_*k*,*ε*_ with *c*_*k*,*ε*′_ position elements. If *c*_*k*,*ε*_ ≥ *c*_*k*,*ε*′_, replace *c*_*k*,*ε*_ with *c*_*k*,*ε*′_ position elements. Finally, a complete binary tree structure is formed where the left node element *c*_*k*,*ε*_ is smaller than the right element *c*_*k*,*ε*′_ at the same level, and ∀*c*_*k*,*ε*_ is larger than its sub-node *c*_*k*−1,*ε*′_ at the previous level.

By searching, the minimum distance is finally moved to the parent node, which is the smallest element min s (in km) in the interval distance heap sorting base vector **S**_*m*_, and this is the optimal distance solution. The children nodes other than this optimal solution are selected from the smallest to the largest according to the ranking rule of the replacement algorithm, and the corresponding children nodes are suboptimal solutions.

**Step 5 .**

Determine the ferry distance index *μ*_1_, bus and subway route index *μ*_2_, cab cost index *μ*_3_, traffic light index *μ*_4_, and congestion index *μ*_5_ between attractions *U*_*z*_ and *U*_*z*+1_.

Starting from the first feature of interest, given the initial value *A*_1_, the iterative value of the motivation output for the motivation subinterval Δ*B*_1_(*U*_1_, *U*_2_) of the attraction route is determined according to the conditions of Step 1 to Step 4.

(7) $$\begin{array}{c} A_{1}^{\prime }=\sum_{g=1}^{5}\mu_{g}A_{1}. \end{array}$$

Then, we have Δ*B*_*z*_(*U*_*z*_, *U*_*z*+1_). The value of the motivational output iteration is

(8) $$\begin{array}{c} A_{z}^{\prime }=\sum_{g=1}^{5}\mu_{g}A_{z}. \end{array}$$

According to Δ*B*_*z*_(*U*_*z*_, *U*_*z*+1_) and Δ*B*_*z*′_(*U*_*z*′_, *U*_*z*′+1_) mutually exclusive and independent relations, the iterative output value of tourist's motivation to visit the final interest feature attraction is

(9) $$\begin{array}{c} A\left(1,U_{t}\right)=\sum_{z=1}^{t-1}\sum_{g=1}^{5}\mu_{g}A_{z}. \end{array}$$

For different elements of the base vector **S**_*m*_ in [*s*_1_, *s*_2_,…, *s*_*γ*_], different iterations of the distance between attractions and different iterations of the corresponding access interval are output. min *A*(1, *U*_*t*_) is taken as the optimal attraction motivation iteration value, which corresponds to the tourist route that can satisfy the maximum motivation benefit of tourists.

## 3. Result Analysis and Discussion

The experiments were conducted on an Intel(R) Core(TM) i7-7700HQ 2.8 GHz CPU, 8 GB RAM, and WINDOWS 10 system using python 3.7. The parameters of the ant colony optimization algorithm are taken as *α* = 4, *β* = 8, *ρ* = 0.7, and *m* = 50. Where *α* is the information heuristic factor. *β* is the expectation heuristic factor. *ρ* is the information volatility factor. *m* is the number of ants.

### 3.1. Analysis of Travel Route Optimization Results

Set a tour group with 20 tourists, planning to start tourism activities in a certain place during the Spring Festival, where there are 20 scenic spots. The 20 scenic spots are numbered, and the corresponding coordinate values are set. The number *A*1 is the departure place of the tourists, which is positioned as (20, 41). The 20 scenic spots are plotted in the same coordinate system, and the corresponding tourist routes are developed. The traditional model and the design model in the text are used to optimize the tourist route and set to reduce the cost of the tour to the minimum value.  Figure 9 presents the scenic distribution map.

The above sample and process were used to complete this experiment, and the shortest travel route is shown in Figure 10. The above experimental results show that the route optimized using the traditional model is significantly longer than the route optimized by the model proposed in the paper under the same number of attractions. The calculation shows that for each additional kilometer of the trip, the fare will increase by 2.5 yuan accordingly. After the route optimization, using the traditional model results will increase the fare by 200 yuan compared to the model optimization results in the paper. The cost for tourists will also increase. At the same time, a survey of tourists shows that tourists disagree with the results of the traditional model optimization.

The time cost of the developed model and other optimization methods were tested and compared to validate the effectiveness further, and the results are displayed in Figure 11. The comparison methods are the traditional model, the GAIG model in the literature [24], the GASA model in the literature [25], the ACOTS model in the literature [26], the SA model, and the IG model.

Figure 11 shows that the proposed model consumes less than 10 s, and the traditional method takes less than 35 s. The proposed model consumes less time and has less time overhead in tour route planning than other existing models. In summary, the optimization results of this paper's model are better than the optimization results of other models. The reasons are as follows: the algorithm in this paper determines the initial path by the greedy algorithm, which can significantly reduce the number of iterations of the algorithm. Due to the existence of ant pheromone, the algorithm in this paper does not search for redundant paths, and the time in finding the optimal path is greatly reduced; the addition of the taboo table better solves the problem that the greedy algorithm is easy to fall into local convergence.

### 3.2. Experimental Analysis of the field of Interest

The data were collected from 100 samples of different occupations, age groups, and education levels across the country by means of an Internet questionnaire, and the data were statistically analyzed to establish the interest field model. According to the actual situation, the tourist groups were divided into middle-aged and old-aged groups, young adults, and children groups. Different groups have different interest needs and distribution of attractions. Based on the age classification and interest distribution, the interest field of each tourist group to the representative attractions in Zhengzhou was established. It builds the convergence model of tourist routes with the interest sites as nodes, determine the best routes, and provide personalized tourist route planning services for tourists.

The feature coding subsets *P*_1_ to *P*_4_ are determined for parks, playgrounds, venues, and leisure consumption in Zhengzhou, which constitute the feature coding set of attractions. Each attraction feature subset contains attraction feature coding elements, as shown in Table 1.

The statistical data are shown in Table 2. The statistical data were applied to construct the interest fields of different tourist groups for the attractions, as shown in Figure 12. *W*_1_, *W*_2_, and *W*_3_ denote the middle-aged and elderly group (*W*_1_), the young adult group (*W*_2_) and the children and adolescents group (*W*_3_), respectively.

From the statistical field of interest of the attractions, it can be seen that the attractions of the park and green areas are the most attractive to the middle-aged and elderly groups, followed by the young adults, and the least attractive to children and teenagers. Amusement parks are the most attractive to children and teenagers, followed by young adults, and less attractive to middle-aged and old people. The attractiveness of each type of venue is comparable to the three types of tourist groups, among which “Zhengzhou Science and Technology Museum” and “Zhengzhou Oceanarium” are the most attractive to children and teenagers. The “Erqi Memorial Hall” is the most attractive to middle-aged and young adults. The interest needs of different groups for each attraction are very different.

A tourist selected the attractions by the smart machine. Because he was not familiar with the attractions in Zhengzhou, he proposed to visit one park and green space, one venue, and one leisure and consumption place in 1 day, according to the travel schedule. The smart machine randomly calls one attraction feature element: ① Bishagang Park *U*_1_*V*_2_, ② Erqi Memorial Museum, *U*_3_*V*_3_, and ③ Erqi Wanda *U*_4_*V*_3_ in each of the four types of attraction feature code subsets and obtains the corresponding codes. The data in Table 3 are obtained by algorithm calculation. The tour order priority is determined based on the iterative values.

From the analysis of the author's algorithm, according to the data in Table 3, the route with the largest iteration value is ②①③. Tourists first visit Erqi Memorial Hall, then visit Bishagang Park, and finally to Erqi Wanda for consumption and entertainment. The whole process can obtain the maximum motivational benefit satisfaction. The next route is ③①②, where tourists first visit Erqi Wanda, then visit Bishagang Park, and finally visit Erqi Memorial Museum, which is the next best motivational benefit satisfaction. The model provides tourists with several optimal and suboptimal routes and explains the planning arrangements of time, itinerary, route, and transportation, respectively. This allows tourists to quickly learn about unfamiliar city tourism information around their own tourism interests and assists them in making rational decisions to obtain the satisfaction of motivational interests.

## 4. Conclusion

In response to the current problems of travel route planning, this paper proposes an on-demand travel route planning model based on improved interest fields. The proposed model combines the advantages of a two-way search algorithm and ant colony algorithm to get rid of the local convergence problem better to improve the greedy algorithm. The shortest path from one attraction to the next attraction is determined using the improved greedy search idea, and the motivation output value covering all interest features is calculated iteratively based on the multinomial access interval iteration index. Finally, the best itinerary is determined to meet the psychological needs of tourists to obtain the maximum motivational benefit satisfaction. The experimental results indicated that the proposed model is consistent with the actual tourism and has strong feasibility and practical significance for intelligent tourism route planning. In real life, tourists may have more than one travel demand to be optimized simultaneously, and how to solve the multiobjective optimization problem of personalized travel route recommendation efficiently will be the next research direction.

## Figures and Tables

**Figure 1:** Area model by the raster method.

**Figure 2:** Location of visitors.

**Figure 3:** Local convergence problem.

**Figure 4:** Comparison of one-way and two-way path search results. (a) One-way search. (b) Two-way search.

**Figure 5:** Two-way search greedy algorithm before and after combining with the ant colony algorithm. (a) Without the ant colony algorithm. (b) With the ant colony algorithm.

**Figure 6:** Spot buffer depth search overlay layer.

**Figure 7:** Depth superposition of distance between road node zones.

**Figure 8:** Complete binary tree composed of base vector **S**_*m*_ elements and their element bits.

**Figure 9:** Scenic distribution map.

**Figure 10:** Shortest route comparison. (a) Result of the proposed model. (b) Result of the traditional model.

**Figure 11:** Time cost comparison.

**Figure 12:** Statistical field of interest by tourist group attractions.

**Table 1:** Subsets of feature codes and their coding elements for attractions.

Subset of attractions	Attraction element code
*P*_1_	*P*_1_ *Q*_1_ People's Park; *P*_1_*Q*_2_ Bishagang Park; *P*_1_*Q*_3_ Zijingshan Park; *P*_1_*Q*_4_ Forest Park; *P*_1_*Q*_5_ Greentown Square; *P*_1_*Q*_6_ Zhengzhou Botanical Garden; *P*_1_*Q*_7_ Zhengzhou Zoo; *P*_1_*Q*_8_ Yellow River Excursion Area

*P*_2_	*P*_2_ *Q*_1_ Century Fun Park; *P*_2_*Q*_2_ Fantasy Fun World; *P*_2_*Q*_3_ Water World *P*_2_*Q*_4_ Children's Park

*P*_3_	*P*_3_ *Q*_1_ Henan Museum; *P*_3_*Q*_2_ Henan Geological Museum; *P*_3_*Q*_3_ Erqi Memorial Museum; *P*_3_*Q*_4_ Zhengzhou Art Museum; *P*_3_*Q*_5_ Zhengzhou Museum; *P*_3_*Q*_6_ Zhengzhou Science and Technology Museum; *P*_3_*Q*_7_ Zhengzhou Oceanarium

*P*_4_	*P*_4_ *Q*_1_ Wangfujing Department Store; *P*_4_*Q*_2_ Department Store; *P*_4_*Q*_3_ Erqi Wanda; *P*_4_*Q*_4_ Zhongyuan Wanda; *P*_4_*Q*_5_ Dehua Pedestrian Street; *P*_4_*Q*_6_ Xiyuan Plaza

**Table 2:** Interest statistics of tourist attractions for different tourist groups.

*P*	*j*	*W*_1_	*W*_2_	*W*_3_
*P*_1_	1	82.32	44.45	20.3
	2	73.54	46.1	43.35
	3	88.35	55.98	30.18
	4	76.28	62.01	30.18
	5	58.72	34.02	23.6
	6	23.05	12.07	13.72
	7	77.38	72.44	80.67
	8	42.26	26.89	12.62

*P*_2_	1	28.54	47.74	93.29
	2	26.34	64.76	93.29
	3	23.05	52.13	86.71
	4	15.37	47.74	97.36

*P*_3_	1	62.78	55.56	30
	2	58.33	47.22	35.56
	3	25.56	31.67	88.33
	4	77.22	77.22	33.33
	5	25.56	32.78	28.89
	6	32.78	55.56	61.67
	7	33.33	65.78	31.81

*P*_4_	1	31.11	88.89	43.89
	2	45	88.33	47.22
	3	35	91.67	47.78
	4	56.11	82.78	34.44

**Table 3:** Tourist-selected attractions and arithmetic data.

Possible routes	①②③	①③②	②①③	②③①	③①②	③②①
Passage interval iteration metrics	0.245	0.223	0.287	0.193	0.228	0.189
	0.201	0.201	0.201	0.201	0.201	0.201
	0.092	0.072	0.092	0.072	0.072	0.07
	0.251	0.168	0.251	0.168	0.168	0.17
	0.13	0.117	0.137	0.122	0.117	0.118
	0.193	0.189	0.223	0.228	0.245	0.245
	0.201	0.201	0.201	0.201	0.201	0.201
	0.072	0.07	0.072	0.072	0.092	0.092
	0.168	0.17	0.168	0.168	0.251	0.251
	0.122	0.118	0.117	0.117	0.13	0.137

Iteration value	0.688	0.578	0.749	0.583	0.715	0.686

## Data Availability

The labeled dataset used to support the findings of this study is available from the corresponding author upon request.
